# Derivation and Verification of the Relationship between Ablation Index and Baseline Impedance

**DOI:** 10.1155/2021/5574125

**Published:** 2021-07-12

**Authors:** Zheng Cai, Sainan Li, Qi Zhang, Chenyuan Wang, Zhen Jin, Ming Fu, Shuai Zhang, Ming Liang, Zulu Wang, Yaling Han

**Affiliations:** ^1^Postgraduate Collage, Jinzhou Medical University, Jinzhou 121000, China; ^2^Department of Cardiology, General Hospital of Northern Theater Command, Shenyang 110016, China

## Abstract

**Objective:**

To explore the quantitative adjustment of ablation index (AI) under different baseline impedance to achieve similar lesion dimensions.

**Methods:**

(1) Keeping the AIs relatively constant, the lesion dimensions in different baseline impedances were studied. (2) According to Joule's law, *Q* = *I*^2^RT, keeping the current (*I*) unchanged, the powers corresponding to different baseline impedances can be obtained. Under different baseline impedances and corresponding powers, the swine hearts were ablated for 30 s in simulated human circumstances. The baseline impedances, the lesion dimensions, and AIs were recorded. And the derivation of empirical formula was achieved according to the AIs and baseline impedance values in similar lesions dimension. (3) Basic AI and baseline impedance (AI_0_/*R*_0_) were set as 400/120 Ω in the common AI groups and 550/120 Ω in the high AI groups, AI values in different baseline impedances were calculated using the empirical formula, and the corresponding lesion dimensions were measured to verify this formula.

**Results:**

(1) Higher baseline impedances were related to smaller lesion dimensions at similar AIs. (2) The lesion dimensions were roughly the same after modulating the baseline impedance and power to keep the electric current relatively constant. The relationship between AI and *R* fitted with experimental data is AI = 1.9933*R* + 203.61 (*r* = 0.9649), and the formula derived is ΔAI = (AI_0_ − 203)/*R*_0_ × Δ*R*. (3) Under the guidance of the empirical formula, there was no significant difference in lesion dimensions between the standard group and the formula guiding groups when AI_0_ = 400, but there was a shrinking tendence when AI > 700.

**Conclusion:**

The lesion depths are negatively correlated with baseline impedance at a certain AI. The relationship between baseline impedance and AI is “ΔAI = (AI_0_ − 203)/*R*_0_ × Δ*R*”. It is verified that when the AI is not too high, the empirical formula can be used to guide the quantitative adjustment of AIs at different baseline impedance, and the lesion depths achieved are roughly the same.

## 1. Introduction

Radiofrequency (RF) catheter ablation has become one of the important treatments for atrial fibrillation (AF), although recurrence after ablation of AF is common [1, 2]. Pulmonary vein electrical reconnection due to the insufficient lesion formation is the main cause of recurrence [2, 3]. There is a close relationship between the lesion dimensions and the ablation success, recurrence, the perioperative complications. Small lesion dimensions may cause recurrence, while large lesion dimensions may damage the adjacent structures and lead to complications. So the prediction and control of lesion dimensions are of great significance in improving RF ablation efficacy and safety.

The tissue damage caused by RF ablation includes resistive-heating damage and conductive-heating damage [4]. It has been reported that the RF lesion was associated with RF time, contact force, and applied power, which were integrated into ablation index (AI) and force-time integral (FTI) [5]. When RF ablation is performed in power-controlled mode in clinical practice, AI is most commonly used to predict the lesion dimensions [5], but the impedance is not counted in the AI calculation formula.

The impedance during ablation is composed of baseline impedance and local impedance. Local impedance is formed by the tissue and blood volume surrounding the ablation catheter, which is relatively consistent. Baseline impedance is generated between the catheter tip and the return patch placed on the patient's skin [6, 7]. During circumferential pulmonary vein ablation for atrial fibrillation, the baseline impedance fluctuates from 100 to 190 Ω, depending on adipose tissue, air, keratinized epidermis, and so on [6]. Difference on impedance may influence the ablation effect at the same AI values. Baseline impedance values and local impedance drops were found helpful to instruct RF delivery or to predict sufficient tissue lesion formation and overheating [4, 7, 8]. The animal studies showed that the lesion dimensions and the baseline impedances were negatively correlated at the same AI values [6]. This study aims to control the lesion depths by controlling current output, to observe the correlation between the baseline impedance and AI under similar lesion depths therefore acquiring the empirical formula, and to verify the reliability of the formula by experiments.

## 2. Materials and Methods

### 2.1. Experimental Preparation and Setting

The protocol for animal experiments in this research was approved by the Institutional Animal Care and Use Committee (IACUC) of the General Hospital of Northern Theater Command. Ten swine hearts bought from a slaughterhouse were used in this research. The smooth myocardium in left ventricular was selected and immersed in a 60 × 40 × 30 cm water bath containing 0.45% solution mixed from 0.9% NaCl solution and purified water, of which the temperature was controlled to 37°C by a heater. The SmartAblate RF generator (Stockert GmbH, Freiburg, Germany) and SmartTouch^TM^ saline-irrigated contact force sensing ablation catheter (Thermocool SmartTouch^TM^, Biosense Webster, CA, USA) were used in power-controlled mode. The catheter was stabilized using an anchor plate and an 8 F sheath and was positioned perpendicular to the myocardial surface during ablation. The schematic diagram is provided in Figure 1. The rate of saline irrigation was controlled to 10 mL/min, the contact force was maintained to 10 g (±2 g), and the power was set to 35 W. The values of baseline impedance were modulated by adjusting the contact area between surface return patch and solution in water bath. The smaller the patch's contact area was, the higher the impedance would be. The AI values, time, power, and impedance during ablation were recorded. The solution in water bath was replaced after every 25 points were ablated. The lesion depths and widths were measured.

### 2.2. Experiment of the Relationship between Baseline Impedance and Lesion Dimension at a Certain AI Value

The in vitro swine hearts were incised along the anterior interventricular groove. The smooth myocardium in left ventricular epicardium was selected and was immersed in 0.45% solution mixed from 0.9% NaCl solution and purified water, of which the temperature was set at 36–37°C. The ST catheter was used and was perpendicular to the myocardium during ablation. The rate of saline irrigation was set at 10 mL/min, pressure at 10 g (±2 g), power at 35 W. The values of basic impedance were modulated by adjusting the contact area between dorsal circular electrode (skin dispersion electrode) and solution in water bath, as well as the distance between catheter and electrode patch. The AI values, time, power, and impedance during ablation were recorded. The solution in water bath was replaced after every 20 points were ablated. The depths and widths of ablation damage ranges were measured.

### 2.3. Experiment of the Relationship between Baseline Impedance and AI at a Certain Lesion Dimension and the Derivation of Empirical Formula

According to Joule's law, *Q* = *I*^2^*RT* (*Q* = heat, I = current, *R* = impedance, *T* = time), the power produced by RF delivery was positively correlated with *I*^2^, impedance, and the duration of RF ablation. The lesion depths were theoretically the same if the current, impedance, and duration were invariant and the heat produced by the ablation catheter was constant [1].

According to formula *P *=* I*^2^*R* (*P* = power), the formula *I*^2^* *=* P*/*R* can be deduced. Keeping the *I*^2^ unchanged, *P*_1__1_/*R*_1_ = *P*_2_/*R*_2_. On the basis of this formula, the corresponding baseline impedance and power of a certain current were calculated as 100 Ω/25 W, 120 Ω/30 W, 140 Ω/35 W, 160 Ω/40 W, and 180 Ω/45 W, which were commonly used in clinical circumstances. After the baseline impedance and power were adjusting to designated values and the catheter was positioned against the cardiac tissue perpendicularly with the contact force at (10 ± 2) g, the ablation was performed on in vitro swine hearts in simulated human circumstances for 30 s at each point. The same RF ablation procedure in each group was repeated for 5 times. After ablation, the lesions were incised, and the depths, widths, and AI values of each lesion were recorded. The mathematical model of baseline impedance and AI was fitted with these data.

### 2.4. Verifying the Reliability of the Formula

The standard AI and the baseline impedance (AI_0_/*R*_0_) were set as 400/120 Ω in the common AI groups and 550/120 Ω in the high AI groups. Baseline impedance was adjusted to different values: 120 Ω, 140 Ω, 160 Ω, 180 Ω, and 200 Ω. The corresponding target AI values were calculated according to the formula derived above. Power was controlled to 35 W. RF energy was applied with the contact force at (10 ± 2) g and did not terminate until the AI reached the target value. The ablation of each group was repeated for 8 times. The AI values, ablation duration, applied power, and impedance during ablation were recorded, and the lesion depths and widths were measured following incision to verify whether the lesion dimensions were consistent.

### 2.5. Statistics

SPSS 26.0 was used for data processing. The differences of lesion dimensions among groups were assessed by ANOVA. The differences of lesion dimensions between the experimental group and the standard group were assessed by independent-sample *T* test. The experimental data of similar lesion depths was inputted into the EXCEL and fitted to curves to acquire the linear relationship between AI and baseline impedance. *P* values were considered statistically significant if < 0.05.

## 3. Results and Discussion

### 3.1. Results

#### 3.1.1. Relationship between Baseline Impedance and Lesion Dimension at a Certain AI Value

When the AI values were about 400 and the baseline impedance was adjusted to 120 Ω, 140 Ω, 160 Ω, 180 Ω, and 200 Ω, the lesion dimensions diminished gradually. The depths decreased from 3.81 mm to 2.61 mm, and the widths deceased from 6.32 mm to 4.98 mm (Figure 2).

#### 3.1.2. Relationship between Baseline Impedance and AI at a Certain Lesion Dimension

After adjusting the baseline impedance and power to keep the I^2^ constant, the lesion depths and widths in different groups with same ablation duration were roughly the same (ablation depths 4.29 ± 0.28 mm, *F* = 1.307,  *P*=0.301; ablation widths 6.37 ± 0.51 mm, *F* = 1.632,  *P*=0.205). There was no significant difference in lesion depths and widths among different groups (Table 1).

#### 3.1.3. The Mathematical Model of Baseline Impedance and AI

The relationship fitted with the recorded AI and impedance data was *y* = 1.9933*x *+* *203.61, *r* = 0.9823 (Figure 3). It could be viewed as AI = *K *×* R* + *b*, so *K *=* *(AI_0_* *−* *203)/*R*_0_ can be deduced. The *K* is positively related to the target ablation depth. The *b* is a constant, which represents the minimum AI value to achieve the target depth when the impedance value is small enough.

According to *K *=* *(AI_0_* *−* *203)/*R*_0_ and AI = *K *×* R* + *b*, it can be derived that

AI* *=* *(AI_0_* *−* *203)/*R*_0_* *×* R *+* *203.

Therefore,

ΔAI* *=* *(AI_0_* *−* *203)/*R*_0_* *×* *Δ*R*.

In order to prove that this formula is still applicable in different ablation depths, the AI_0_ = 400, *R*_0_ = 120 Ω was used as parameters of basic depth to represent the common AI and impedance. Δ*R* means the value of impedance change, and ΔAI means the AI value needing to adjust.

#### 3.1.4. Reliability of the Formula

Under the guidance of the empirical formula, the AI values of corresponding baseline impedance at 140 Ω, 160 Ω, 180 Ω, and 200 Ω in both the common AI groups and the high AI groups were calculated and ablation was performed. The lesion depths in the common AI groups were roughly the same and there was no significant difference (Figures 4 and 5 and Table 2). However, in the high AI groups, when AIs were 550, 608, and 666, the lesion depths were very similar, and there is no significant difference. But when the AIs were 723 and 781, the lesion depths had the shrinking tendence compared with the control group (AI_0_ = 550), though no significant difference was seen when AI was 723 (Figure 6, Tables 3 and 4).

### 3.2. Discussion

AI is often clinically used to guide RF catheter ablation of circumferential pulmonary vein isolation (PVI) for AF. AI integrates applied power, contact force, and ablation duration and can predict the lesion dimension prospectively and accurately [9, 10]. The application of AI has significantly improved the acute success rate of ablation and decreased the ablation duration as well as the incidence of complication and recurrence [5]. However, during PVI for AF, the baseline impedance of human body sometimes fluctuates heavily [6]. The AI formula does not take into consideration the influence of impedance changes on the ablation results. In this research on the relationship of AI, baseline impedance, and lesion dimensions, there were 3 main findings. (1) The lesion depths are negatively correlated with baseline impedance at a certain AI. (2) The relationship between baseline impedance and AI is “ΔAI* *=* *(AI_0_ − 203)/*R*_0_ × Δ*R*”. (3) It is verified that when the AI is no more 700, the empirical formula can be used to guide the quantitative adjustment of AI at different baseline impedance, and the lesion depths achieved are relatively equal. These findings would be helpful for instructing the parameter adjustment in clinical situation.

During circumferential PVI for AF, the thickness of different sites in pulmonary ostia is different, ranging from 0.7 mm to 4.3 mm, and the esophagus is close to the left atrial posterior wall in most patients, especially during left superior pulmonary vein ablation [11]. So more accurate lesion prediction and energy adjustment are very important during AF ablation to create proper lesion dimensions with safety at different part of left atrium.

The negative relationship between baseline impedance and lesion dimensions at a certain AI value found in our research is consistent with the results from Barkagan and his colleagues [6]. As we all know, the current delivered to the ablative tissue depends on the local impedance during ablation and its proportion to the total impedance. Since the local impedance is relatively constant in the absence of change in tissue-catheter tip interface and contact force, the increase in baseline impedance will lead to the decreased proportion of local impedance, thus the current delivery to the ablation site is diminished and the lesion dimension decreases [6]. Therefore, when the baseline impedance increases but the AI value is not adjusted accordingly, RF ablation may fail to achieve the target ablation depths. And when baseline impedance decreases but the AI value is not adjusted accordingly, the lesion dimensions may be excessive, increasing the probability of complications [12].

Under the condition of high baseline impedance, increasing the number of surface return patches or repositioning the patches from the standard position above the left thigh muscle to the low impedance area with less subcutaneous adipose tissue between the left ilium and the chest cavity can reduce the impedance to the normal range to make the ablation more efficient and reduce complications during ablation [7, 13]. However, still sometimes the impedance remains high even by adjusting the return patch. Thus, ablation at high baseline impedance would still be a challenge for operators.

When the target AI is not too high, the empirical formula derived in this research can be used to guide the quantitative adjustment of AI to different baseline impedance, so that similar lesion dimensions can still be achieved in spite of different baseline impedances. So in special baseline impedance conditions, operators can adjust the AI value instead of adjusting the baseline impedance to achieve the target lesion dimension. The lesion dimensions during formula verification fluctuated slightly, but with no significant difference. The main reasons of data fluctuations may include catheter contact force fluctuations, solution concentration change caused by catheter irrigation during ablation, and accidental error. However, when the target AI is too high, such as 723 and 781 in this research, the lesion depths had the shrinking tendence, though no significant difference was seen when AI was 723, which might be related to the small sample size. We thought the deviation at high AI values might be due to the upper limit of the AI calculation formula at 650. When the AI value is above this limit, the AIs may not accurately predict the lesion dimension. Due to the limitation of AI calculation formula, the applicability of the empirical formula derived from our research may also be limited. The empirical formula is applicable only when the AI is no more than 650. Fortunately, the condition of target AIs exceeding 650 is very rare in clinical practice. And when this happens, operators should decease the baseline impedance by increasing the number of surface return patches or repositioning it to the low impedance area to reduce the baseline impedance, as we mentioned above. When the baseline impedance is reduced, the target AIs will be correspondingly decreased as well.

## 4. Limitation

In the early stage of fitting formula, we took a large impedance span (20 Ω) and a relatively small sample of data, so the data used to fit the formula may be biased. In addition, the solution we used was different from the blood media in in vivo animal experiments or actual clinical conditions, so the empirical formula derived may not be fully consistent with the clinical practice.

## 5. Conclusions

The lesion dimensions are negatively correlated with baseline impedance at a certain AI value. The relationship between baseline impedance and AI is in accordance with ΔAI* *=* *(AI_0_ − 203)/*R*_0_ × Δ*R*. It is verified that when the AI is not too high the empirical formula can be used to guide the quantitative adjustment of AI at different baseline impedance, and the lesion depths achieved are roughly the same.

## Figures and Tables

**Figure 1:** Schematic diagram of the in vitro ablation model.

**Figure 2:** The lesion dimensions in increased baseline impedance and similar AI.

**Figure 3:** The relationship between the AI and the baseline impedance in the similar ablation depths.

**Figure 4:** The lesion depths, baseline impedance, and AI values in formula-guided ablation in the common AI groups.

**Figure 5:** The variation tendency of lesion dimensions in the common AI groups.

**Figure 6:** Baseline impedance and AI values in the high AI groups and the corresponding lesions created under these settings.

**Table 1:** The relationship among different basic impedance, power, and the ranges of ablation damage when the current and pressure were relatively constant.

Impedance (Ω)	Power (W)	AI	Average pressure (g)	Depths (mm)	Widths (mm)
99.0 ± 1.0	25	392.6 ± 6.9	10.0 ± 1.0	4.13 ± 0.28	6.40 ± 0.20
119.8 ± 1.5	30	452.2 ± 7.8	11.2 ± 0.8	4.14 ± 0.24	6.57 ± 0.90
140.4 ± 0.9	35	486.2 ± 12.6	11.0 ± 1.0	4.41 ± 0.23	6.68 ± 0.30
159.2 ± 1.6	40	519.6 ± 10.0	10.6 ± 0.5	4.38 ± 0.32	6.01 ± 0.44
180.0 ± 0.0	45	559.6 ± 11.3	11.0 ± 1.0	4.37 ± 0.28	6.17 ± 0.23

AI = Ablation index.

**Table 2:** The target AI, actual AI, and damage ranges obtained in different impedance under the guidance of empirical formula.

Impedance (Ω)	Target AI	Actual AI	Depths (mm)	Widths (mm)
120.0 ± 1.1	400	402.4 ± 1.6	3.70 ± 0.35	6.30 ± 0.33
140.0 ± 0.5	433	433.6 ± 2.4	3.81 ± 0.43	6.07 ± 0.30
159.9 ± 0.4	466	463.4 ± 2.6	3.85 ± 0.35	6.11 ± 0.38
179.9 ± 0.8	499	497.6 ± 1.7	3.87 ± 0.20	6.18 ± 0.38
200.4 ± 0.7	531	533.9 ± 1.6	3.82 ± 0.22	6.09 ± 0.55

**Table 3:** The lesion depths in the high AI groups and the *P* values between the experimental groups and control group.

	550/120 Ω	608/140 Ω	666/160 Ω	723/180 Ω	781/200 Ω
Depths (mm)	5.778 ± 0.282	5.766 ± 0.205	5.778 ± 0.452	5.472 ± 0.395	5.23 ± 0.325
*P* values		0.941	1	0.196	0.022

**Table 4:** The lesion widths in the high AI groups and the *P* values between the experimental groups and control group.

	550/120 Ω	608/140 Ω	666/160 Ω	723/180 Ω	781/200 Ω
Widths (mm)	10.002 ± 0.401	9.308 ± 0.506	9.486 ± 0.581	8.198 ± 0.470	8.436 ± 0.674
*P* values		0.053	0.141	0.000	0.002

## Data Availability

The statistical and image data used to support the finding of this study are included within the article.
